RETRACTED

# Toxic and repellent impacts of botanical oils against *Callosobruchus maculatus* (Bruchidae: Coleoptera) in stored cowpea [*Vigna unguiculata* (L.) Walp.]

**DOI:** 10.1371/journal.pone.0267987

**Published:** 2022-05-23

**Authors:** Muhammad Shahid Nisar, Shahbaz Ali, Tassaduq Hussain, Hassan Ramzan, Yasir Niaz, Inzamam Ul Haq, Faiza Akhtar, Mona S. Alwahibi, Mohamed S. Elshikh, Hazem M. Kalaji, Arkadiusz Telesiński, Mohamed A. A. Ahmed, Marwa I. Mackled

**Affiliations:** 1 Department of Plant Protection, Faculty of Agricultural Sciences, Ghazi University, Dera Ghazi Khan, Pakistan; 2 Department of Agricultural Engineering, Khwaja Fareed University of Engineering and Information Technology, Rahim Yar Khan, Punjab, Pakistan; 3 Department of Zoology, Ghazi University, Dera Ghazi Khan, Pakistan; 4 College of Plant Protection, Gansu Agricultural University, Lanzhou, Lanzhou, China; 5 Department of Environmental Sciences, Faculty of Life Sciences, Balochistan University of Information Technology Engineering and Management Sciences, Quetta, Balochistan, Pakistan; 6 Department of Botany and Microbiology, College of Science, King Saud University, Riyadh, Saudi Arabia; 7 Department of Plant Physiology, Institute of Biology, Warsaw University of Life Sciences SGGW, Warsaw, Poland; 8 Institute of Technology and Life Sciences - National Research Institute, Falenty, Raszyn, Poland; 9 Department of Bioengineering, West Pomeranian University of Technology in Szczecin, Szczecin, Poland; 10 Plant Production Department (Horticulture - Medicinal and Aromatic Plants), Faculty of Agriculture (Saba Basha), Alexandria University, Alexandria, Egypt; 11 Department of Stored Product Pests, Plant Protection Institute, Agriculture Research Center (ARC), Sabahia, Alexandria, Egypt; Anhui Agricultural University, CHINA

## Abstract

Cowpea (*Vigna unguiculata*) is an important legume which is consumed globally for protein intake, particularly in Asian states. It is a well-known source of dietary fiber, protein, minerals, and vitamins. The cowpea grains are stored after harvest and used till the next harvest. However, the grains are infested by storage pests, primarily *Callosobruchus maculatus*. Hence, effective management strategies are needed to protect the stored grains form the pests. This study assessed the efficacy of some edible oils in suppressing *C*. *maculatus* infestation in stored cowpea grains. Four different botanical oils (i.e., mustard, neem, poppy, and pumpkin) at four different concentrations (i.e., 0.5, 1.0, 1.5 and 2.0 ml per 100 g grain) were included in the study. A control treatment without any botanical oil was also included for comparison. The relevant concentrations of botanical oils were poured into plastic containers containing 100 g cowpea grains and ten *C*. *maculatus* adults were released. The jars were sealed and placed at room temperature. Data relating to mortality, oviposition, F1 adult emergence, and seed weight loss were recorded. The tested botanical oils and their concentrations significantly affected mortality after one day. Mortality after 2^nd^ and 3^rd^ days remained unaffected by botanical oils and their different concentrations. The highest mortality was recorded in neem oil-treated grains followed by poppy, pumpkin, and mustard oils. Increased oviposition rate was observed in the grains treated with mustard and pumpkin oils, while those treated with neem and poppy oil recorded decreased oviposition. The control treatment had increased oviposition rate compared to tested botanical oils. All botanical oils significantly inhibited egg laying percentage. The highest germination was recorded for the grains treated with mustard oil followed by pumpkin, poppy, and neem oils, respectively. The lowest germination was recorded for control treatment. Significant differences were noted for *C*. *maculatus* repellency among botanical oils. No emergence of adults (F1 progeny) was recorded in all tested botanical oils; thus, F1 progeny was inhibited by 100%. Weight loss, damage percentage, and holes in the grains were not recorded since F1 progeny did not emerge. It is concluded that tested botanical oils are promising and could be utilized to control *C*. *maculatus* in cowpea grains during storage.

RETRACTED

## Introduction

Cowpea [*Vigna unguiculata* (L.) Walp.] is an important crop in the conventional cultivation systems of semi-arid areas in Africa, Asia, and southern and central America. It is known by various common names such as asparagus bean, black eye bean, China pea, Kaffir bean, southern pea, black eye pea, lobia, and yard long bean in different countries of the world. Cowpea has multiple uses since fresh leaves, green seeds, and green seed pods are utilized as vegetable, while dry seeds are used in the preparation of different foods [1]. Cowpea serves as a nutritive fodder for livestock. The protein content in the leaves and grains of cowpea in crude form varies from 22 to 30%) on dry weight basis. The cowpea stalk contains 13–17% protein with increased digestion and decreased fiber extent [2].

Cowpea is cultivated in rainfed areas for several purposes, i.e., grains, fodder, vegetable, green manure, regulating soil fertility and as a cover crop to decrease water loss through evaporation. Sebetha et al. [3] reported that cowpea contains abundant protein content (22 to 33%), 53.56 to 57.36% carbohydrates and decreased anti-nutritious extent compared to common beans. Cowpea is cultivated under climate extremes, such as drought-prone areas and mostly on alkaline soils. It cannot resist frost and heat stress significantly decreases its development [4].

RETRACTED

Generally, Pakistani soils are less fertile and lack nitrogen (N). The use of N fertilizer is decreasing in Pakistan due to high price, low availability of credit, and unavailability at suitable time. Therefore, legumes must be included in the cropping systems because they can increase soil N level by atmospheric nitrogen fixation [5]. It is known that legumes fix 50 to 100 kg N per hectare [6]. Low accessibility of green fodder is the major reason of low livestock production in Pakistan, and availability is reduced by 75% during feed shortage [7]. Leguminous fodder is essential in livestock production because of high calcium, minerals, proteins, vitamins, and phosphorus [8].

Essential oils and extracts of different plants species are a promising alternative to insecticides for insect pest management. Bio-insecticides are naturally occurring insecticides extracted from plants and include a variety of bio-active compounds [9, 10]. The plant extracts may suppress various insects based on their physiological features and plant tye. Extracts and essential oils of plants exert ovicidal and larvicidal effects on insects, inhibit respiration, suppress oviposition, act as antifeedants, repellents, attractants, reduce adult emergence and hinder host plants identification [11–14]. Many essential oils repel insects due to their repellent materials which affect smell, taste, and touch senses of the target insects. Usually, repellents prevent insects from reaching their targets [15–17].

*Azadirachta indica* is one of the most known species serving as toxic bio-insecticide in pest management. Several studies have reported that various plants species exert harmful impact on egg-laying, fecundity, and feeding capacities of various insect species, suppress the growth of larvae, pupae and adult, and increase mortality [18–21].

Poppyseed oil (*Papaver somniferum*: Papaveraceae) is an eatable oil taken from opium seeds. Poppy oil is edible and have medicinal uses. It is used in the manufacturing of soap, paint, and varnish. Poppy seeds contain higher amounts of vitamin E, palatable, and lack narcotic characteristics with an oil yield of 45 to 50% [18].

Mustard (*Brassica campestris* L.) oil is naturally repellent due to the presence of linoleic acid, allyl-isothiocyanate, erucic acid and oleic acid [22]. Mustard oil is utilized in two forms, i.e., essential oil and fat comprised vegetable oil [23].

Pumpkin is highly nutritious and contains better grade oil, serves as a good protein source, and possesses antioxidant and medicinal properties (anti-fungal, anti-bacterial, anti-diabetic and anti-inflammation). Pumpkin seeds have been utilized to extract oil and pharmacological purposes since ancient times [24].

RETRACTED

Like other pulses, cowpea is infested by storage insect pests. Insect pests’ infestations significantly decreases cowpea yield, seed quality, and profitability. Although it is a short duration crop, numerous insect pests damage cowpea after germination till harvest, which lower productivity. Nevertheless, few pests infest grains during storage. The most important pest during storage cowpea bruchid (*C*. *maculatus* F.). It is a significant pest of legumes in Asian and African countries during storage. The larvae of the pest bore into grains and consume endosperms; thus, making seeds unfit for consumption and germination [25]. The pupae develop inside the grains, while adults emerge through grain holes [16]. The *C*. *maculatus* infests 50–90% stored cowpea annually in tropical Africa. Mbaiguinam et al. [26] reported that highest cowpea infestation (100%) in the conventional stored method is common within three to five months.

Application of insecticides is the commonly used method to protect stored grains from pest infestation. However, high prices, unavailability to the small scale farmers, residual impacts, pest resistance, persistence, and detrimental effects on non-target organisms make insecticides an unattractive option [27]. Therefore, novel insecticides with new modes of action and low residual impacts are needed. Therefore, several researchers are looking towards natural products, specifically edible plant species, as resources of degradable insecticides which are safe for human and the environment [28]. This study was aimed at testing the efficacy of some botanical oils (mustard, neem, poppy, and pumpkin) against *C*. *maculatus*. Adult mortality, oviposition, and F1 progeny emergence from stored cowpea were recorded.

## Materials and methods

This study was conducted in Zoology laboratory (30.039469 ºN, 70.634441 ºE) at Ghazi University, Dera Ghazi Khan, Pakistan. No ethical permissions were required for the study as no endangered species were involved.

### *Callosobruchus maculatus* culture

The *C*. *maculatus* is the most damaging pest of pulse crops. Cowpea grains were procured from local grain market of Dera Ghazi Khan, Pakistan (30.037352 ºN, 70.649772 ºE). The grains (500 g) were placed in a plastic jar (1 kg capacity) and thirty *C*. *maculatus* adults (equal ratio of males and females) were released in the jar. The jar was covered with muslin cloth by a rubber band. Oviposition started after ten days and then males and females were separated. The new adults emerged 25 days after oviposition which were used in this experiment. The plastic jar was kept under 27–32 ºC temperature and 65–70% relative humidity.

RETRACTED

### Bioassay

Four different oils were tested for their efficacy against *C*. *maculatus*. Four different concentrations of each oil, i.e., 0.50, 1.00, 1.50 and 2.00 ml along with an untreated (0.00 ml) control were used. A total 100 g cowpea grains were placed plastic jars and different concentration of the oils were poured into the jars containing health grains. Ten adults (5 males and 5 females) were released in the jars containing healthy grains and relative concentration of the tested oils. The jars were covered with muslin cloth by a rubber band. The treatments were arranged in a completely randomized design (CRD) with three replications.

### Data collection

Data relating to adult mortality, total mortality, mortality percentage, oviposition, oviposition inhibition percentage, hatching percentage, F1 progeny, F1 progeny reduction percentage, male and female count, number of holes, seeds weight loss percentage, seed damage percentage, repellency and germination percentage were recorded.

The adult mortality was observed 24, 48, and 72 hours after the release of the adults in the jars. Mortality was observed by touching the *C*. *maculatus* abdomen with the help of a camel hairbrush. When they adults did not move upon touching, they were considered as dead. The dead adults were separated and removed from the jars. The total mortality was computed by collecting dead adults after 24, 48, and 72 hours. Percent mortality was computed by the following formula.


$$\text{Mortality}\;\left(\text{\%}\right)=\frac{Number\;of\;dead\;adults}{Total\;number\;of\;adults\;released}\times 100$$

The mean daily mortality was calculated by using the formula given below.


$$\text{Mean}\;\text{daily}\;\text{mortality}=\frac{Number\;of\;dead\;adults}{Total\;number\;of\;observation\;days}$$

After mortality observation, all dead and live adults were removed from the jars and eggs deposited on the cowpea grains were counted with the help of a magnifying lens. The oviposition inhibition percentage was computed by the formula given below.


$$\text{Oviposition}\;\text{inhibition}\;\text{\%}=\frac{Egg\;count\;in\;control\;treatment}{Egg\;count\;in\;relevant\;treatment-Egg\;count\;in\;control\;treatment}\times 100$$

All emerged adults twenty-five days after oviposition were counted from all treatments to record F1 progeny. The reduction percentage in F1 progeny was computed by the below equation.


$$\text{F}1\;\text{progeny}\;\text{reduction}\;\text{\%}=\frac{Number\;of\;emerged\;adults\;in\;treatment-Number\;of\;emerged\;adults\;in\;control}{Number\;of\;emerged\;adults\;in\;control}\times 100$$

A total 50 grains were randomly selected from all treatments after adult emergence, checked carefully, and number of holes present on each grain were counted. For calculating damage percentage, 20 grains were randomly selected from each treatment and holes-carrying grains, or damaged grains were counted. The percent damage was computed by unitary method. The grains in all treatments were weighed at the start and end of the treatment periods. The weight loss percentage was computed by unitary method. Seed germination of ten randomly selected cowpea seeds from all treatment was recorded in Petri dishes and percent germination was computed. Repellency percentage was computed by the formula given below.


$$\text{Repellency}\;\left(\text{\%}\right)=\frac{\text{NC}-\text{NT}}{\text{NC}+\text{NT}}\times 100$$

Repellency bioassay comprised two plastic jars (750 ml) joined at rims with nylon mesh tube. A 100 g cowpea grains treated with specific concentration of tested oils were inserted into the plastic jar at one endpoint of a tube having control grains on the other end. Five pairs (10 adults) were released into the mesh tube with a round hole at the center of the tube. The repellency was assessed after 40 minutes of insect inoculation.

RETRACTED

### Statistical analysis

The collected data were statistically analyzed by using analysis of variance (ANOVA), and Duncan’s multiple range post-hoc test 5% was probability was to compare treatments’ means. The data used to prepare this manuscript are given S1 Dataset.

## Results

Highly significant differences were recorded among tested botanical oils and their concentrations as for mortality after 1^st^ day (Fig 1a). The mortality increased with increasing concentration of all oils and the highest concentration (2.0 ml) resulted in the highest mortality. The neem, poppy, and pumpkin oils resulted in higher mortality compared to mustard oil. Statistically similar results were recorded for mustard (2.0 ml), neem (1.0 ml), poppy (1.0 ml), and pumpkin (1.5 ml) oils (Table 1).

**Fig 1:** The impact of different botanical oils and their concentrations on *C*. *maculatus* mortality at 1^st^ (a), 2^nd^ (b) and 3^rd^ day (c) and total mortality (d).

**Table 1:** The impact of different botanical oils and their concentrations on *C*. *maculatus* mortality at different time intervals and total and percentage mortality.

Treatments	Mortality on 1^st^ day	Mortality on 2^nd^ day	Mortality on 3^rd^ day	Total mortality	Total mortality %
**Botanical oils**					
Mustard oil	3.80±2.91	2.73±1.58	1.07±1.39	7.60±3.85	76.00 ±38.51
Neem oil	5.93±3.47	1.73±1.44	0.40±0.74	8.07±4.01	80.67±40.08
Poppy oil	5.20±3.36	2.20±1.57	0.47±0.83	7.93±3.95	79.33±39.55
Pumpkin oil	4.80±3.00	2.60±1.68	0.47±0.74	7.87±3.94	78.67±39.44
**Concentrations**					
0 ml	0.00±0.00	0.00±0.00	0.33±0.49	0.33±0.49	3.33±4.92
0.5 ml	3.17±1.47	3.92±0.79	2.17±0.83	9.25±0.96	92.5±9.65
1.0 ml	5.92±1.24	3.42±0.79	0.42±0.79	9.83±0.39	98.33±3.89
1.5 ml	7.25±1.14	2.58±0.90	0.08±0.29	9.92±0.28	99.17±2.89
2.0 ml	8.33±0.89	1.67±0.89	0.00±0.00	10.00±0.00	100.00±0.00

Different oils and their concentrations resulted in statistically similar mortality after 2^nd^ day (Fig 1b). Table 1 for mean comparison depicted that the highest mortality was observed with poppy (0.5 ml), mustard (0.5 ml) and pumpkin (0.5 ml) oils, while no mortality was recorded in the control treatment. Non-significant variations in the mortality after 3^rd^ day were noted among various oil concentrations (Fig 1c). The increased mortality was recorded with mustard (0.5 ml). The control treatment represented 0.33% mortality after three days (Table 1). Total mortality demonstrated statistical similarity among all oil treatments (Fig 1d). Mean comparison for total mortality depicted that mustard oil-treated grains recorded the lowest mortality, whereas grains treated with neem, poppy and pumpkin oils recorded higher mortality (Table 1).

RETRACTED

Different oils and their concentrations had non-significant effect on percent mortality (Fig 2). Mean comparing depicted that all oils caused significant mortality. Higher mortality was recorded with neem oil, whereas lower mortality was observed in mustard oil-treated grains. Only 3.33% mortality was recorded in control (0 ml) grains.

**Fig 2:** The impact of different botanical oils and their concentrations on percent mortality of *C*. *maculatus*.

Significant variations were recorded among tested oils and their concentrations for oviposition (Fig 3a). A decrease in oviposition was recorded in neem oil-treated grains. The oviposition was statistically similar in mustard (2.0 ml), neem (1.0 ml), poppy (1.0 ml) and pumpkin (1.5 ml) oils. Higher oviposition was observed in control treatment followed by mustard oil-treated grains at 0.5 ml, while neem oil-treated grains at 2.0 ml recorded the lowest oviposition (Table 2).

**Fig 3:** The impact of different botanical oils and their concentrations on oviposition (a), oviposition inhibition % (b), hatching (c), and F1 progeny (d) of *C*. *maculatus*.

**Table 2:** The impact of different botanical oils and their concentrations on oviposition, oviposition inhibition, hatching, F1 progeny and F1 progeny reduction of *C*. *maculatus*.

Treatments	Oviposition	Oviposition inhibition %	Hatching	F1 progeny	F1 progeny reduction %
**Botanical oils**					
Mustard oil	89.80±76.73	60.43±33.79	15.06±31.20	34.2±70.83	80.00±41.40
Neem oil	63.27±86.41	72.12±38.05	15.06±31.20	34.2±70.83	80.00±41.40
Poppy oil	68.07±84.12	70.01±37.04	15.06±31.20	34.2±70.83	80.00±41.40
Pumpkin oil	77.33±82.10	65.92±36.16	15.06±31.20	34.2±70.83	80.00±41.40
**Concentrations**					
0 ml	22.70±3.41	0.00±0.00	75.32±2.09	171.00±4.74	0.00 ± 0.00
0.5 ml	76.67±22.65	66.22±9.98	0.00 ± 0.00	0.00 ± 0.00	100.00 ± 0.00
1.0 ml	33.33±15.71	85.30±6.91	0.00 ± 0.00	0.00 ± 0.00	100.00 ± 0.00
1.5 ml	22.17±10.12	90.23±4.45	0.00 ± 0.00	0.00 ± 0.00	100.00 ± 0.00
2.0 ml	13.92 ±6.99	93.86±3.08	0.00 ± 0.00	0.00 ± 0.00	100.00 ± 0.00

Highly significant difference was noticed in botanical oils and their concentrations for oviposition inhibition (Table 2). Different treatments, i.e., neem (2.0 ml), pumpkin (0.5 ml), mustard (0.5 ml), and control (0.0 ml) significantly differed from each other, while remaining treatments were non-significant (Fig 3b).

RETRACTED

Hatching and emergence of F1 progeny was not observed in all botanical oils-treated grains (Fig 3c and 3d). However, F1 progeny (171%) was recorded in the control treatment (Table 2).

Due to non-emergence of adults from the botanical oils-treated grains, all botanical oils exhibited their potency towards *C*. *maculatus* (adults). Hundred percent first progeny reduction was recorded in all botanical oils (Fig 4, Table 2).

**Fig 4:** The impact of different botanical oils and their concentrations on F1 progeny reduction of *C*. *maculatus*.

Significant number of holes in grains were recorded for control treatment (38.33), whereas no holes were noted on the grains reacted with all tested oils (Fig 5a). Grains treated with different oils did not exhibit any weight loss, whereas control treatment recorded 23.33% loss in grain weight (Fig 5b, Table 3). No damage was observed in grains treated by various oils at different concentrations. However, 60% grains in the control treatment were damaged by the pest infestation (Fig 5c, Table 3).

**Fig 5:** The impact of different botanical oils and their concentrations on holes count (a), weight loss (b) and damage caused (c) by *C*. *maculatus*.

**Table 3:** The impact of different botanical oils and their concentrations on holes count, weight loss % and damage % of *C*. *maculatus*.

Treatments	Holes count	Weight loss (%)	Damage (%)
**Botanical oils**			
Mustard oil	7.67±15.91	4.67±9.67	12.00±24.85
Neem oil	7.67±15.91	4.67±9.67	12.00±24.85
Poppy oil	7.67±15.91	4.67±9.67	12.00±24.85
Pumpkin oil	7.67±15.91	4.67±9.67	12.00±24.85
**Concentrations**			
0 ml	38.33±2.60	23.33±1.30	60.00±1.75
0.5 ml	0.00 ± 0.00	0.00 ± 0.00	0.00 ± 0.00
1.0 ml	0.00 ± 0.00	0.00 ± 0.00	0.00 ± 0.00
1.5 ml	0.00 ± 0.00	0.00 ± 0.00	0.00 ± 0.00
2.0 ml	0.00 ± 0.00	0.00 ± 0.00	0.00 ± 0.00

Significant differences were noted in the seed germination of grains treated with different oils (Fig 6a). The highest seed germination was observed in mustard (0.5 ml) and pumpkin (0.5 ml) oils, respectively. However, the lowest seed germination was recorded for the seeds treated with neem oil (2.0 ml). Control treatment represented 33.33% seed germination. The reduced concentration of botanical oils showed increased germination ability (Table 4).

RETRACTED

**Fig 6:** The impact of different botanical oils and their concentrations on germination and repellency.

**Table 4:** The impact of different botanical oils and their concentrations on germination and repellency.

Treatments	Germination (%)	Repellency (%)
**Botanical oils**		
Mustard oil	74.66±23.25	45.33±32.48
Neem oil	53.33±19.14	72.00±39.13
Poppy oil	65.33±17.67	61.33±35.83
Pumpkin oil	69.33±21.20	57.33±33.69
**Concentrations**		
0 ml	33.33±4.92	0.00±0.00
0.5 ml	85.83±9.00	51.67±19.92
1.0 ml	80.00±9.53	70.00±17.09
1.5 ml	69.16±13.11	81.66±15.85
2.0 ml	60.00±15.37	93.33±9.84

Data relating to repellency revealed significant variations among botanical oils (Fig 6b). The increased repellent influence was noticed with neem oil at 1.5 and 2.0 ml, while decreased repellency was demonstrated by mustard oil (0.5 ml). Statistically same repellency was observed for the seeds treated with poppy and pumpkin oils at 2.0 ml as same as mustard oil (2.0 ml), neem oil (1.0 ml) and poppy oil (1.5 ml), and neem oil (0.5 ml) with poppy oil (1.0 ml) and pumpkin oil (1.5 ml) (Table 4).

## Discussion

The neem, poppy, pumpkin, and mustard oils at various concentrations were used in the current study to test their efficacy in suppressing *C*. *maculatus* infesting cowpea grains. Regnault-Roger, [29] stated that various botanical products (powdered, extract, and oil forms) might be utilized as fumigants, topical potents, repellents, antifeedants, and progeny inhabitants. The botanical oils caused significant mortality after one day of application in the current study. Paneru and Shivakoti [30] reported that *A*. *calamus* (rhizome powder), ash of rice husk and *Brassica spp*. (mustard) oil caused significant mortality of *C*. *maculatus* after seven days when used at 0.5, 1, and 2% formulations. For two days neem oil caused 100% mortality in *C*. *maculatus*. These results correspond to the findings of present study where 100% adult mortality of *C*. *maculatus* was observed. Chelav and Khashaveh [31] stated that an increased mortality was recorded with 10 ml poppy oil per kg of grains after three days exposure. In our study, an increased mortality was observed by neem oil followed by poppy oil at 2.0 ml concentration per 100 g grains with three days exposure. Neem oil contains azadirachtin, which is highly potent against *C*. *maculatus*.Ahmed et al. [32] stated that 100% mortality of *C*. *chinensis* was achieved within three days. Sousa et al. [33] assessed the comparative potency of mustard essential oil against *C*. *maculatus* and *Sitophilus zeamais* life stages (old and young larval stage, pupal, and adult stage) by using formulation response bioassays. The findings expressed that various life stages of both insects behaved differently against mustard essential oil and adults were highly susceptible compared to immature phases.

RETRACTED

Wahedi et al. [34] stated neem seed oil as the main potent for *C*. *maculatus* adults and also decrease the egg-laying ability of females. This is in line with our investigation as the lowest egg-laying (oviposition) was observed in grains treated with neem oil followed by poppy, pumpkin, and mustard oils. Mbaiguinam et al. [26] also reported that neem oil is effective in suppressing populations of different insects. Ilesanmi and Gungula [35] investigated the potentials of neem and *Moringa oleifera* (moringa) seeds against storage ability of cowpea and reported that neem (0.5 ml per 200 g) treated grains contained minimum eggs count.

In the case of oviposition, the present study demonstrates that neem oil was a significant inhibitor of egg-laying followed by poppy, pumpkin, and mustard oils. This was in accordance with Jagjeet et al. [36] who stated that oils’ application decreased egg-laying of insects. Ojebode et al. [37] reported about the potent potential of orange peel (*Citrus sinensis*), lemongrass (*Cymbopogon citratus*), and neem in two forms (extracts and oils) on *C*. *maculatus*. All products were potent against the adults and restricted hatching. Gupta and Apte [38] reported the efficacy of neem against *C*. *maculatus* seed infestation, oviposition, holes making, weight deficit, and mean growth period. Abd El-Aziz, [39] stated eucalyptus and clove oil as egg-laying inhibitors of *C*. *maculatus*. In our study, the lowest oviposition, intact seeds, and weight deficit was noticed in neem oil-reacted grains. Ketker [40] assessed the castor, neem, and coconut oils toward pulse bruchid in green gram and finally reported neem oil as the best surface protector. Neem oil provided the egg laying deterrence with suppressing insects.

In the current study no adults emerged from the grains treated with tested oils. Ramzan [41] stated that mustard oil significantly inhibited the emergence of *C*. *maculatus* adults. Ahmed et al. [42]observed that sesame and neem oils completely hindered the emergence of *C*. *chinensis* adults. Ismail [43] reported that cotton leafworm larvae were suppressed by orange, sesame, camphor, pepper and pumpkin.

RETRACTED

Since no adults emerged from the grains treated with different oils in the present study, no weight loss, damage, and holed grains were recorded. Parmar and Patel [44] reported that mustard oil protected the and green gram against storage insect infestation. Khalequzzaman et al. [45] revealed that groundnut oil completely suppressed progeny emergence and decreased grain weight reduction. Thakur and Pathania, [46] reported a 100% mortality by pepper, neem and mustard oils seven days after exposure. Kobir et al.[47] stated that increased rate of mustard (3 ml) and coconut (4 ml) oils resulted in decreased weight reduction and seed infestation after one month. Lale et al. [48] determined the potency of neem oil against egg-laying rate, progeny, and infestation of *C*. *maculatus* in cowpea grains and stated that it was highly effective. Manju et al, [49] observed the potential of oils in the sequence of citronella oil ˃ geranium oil ˃ mint oil ˃ mustard oil ˃ coconut oil ˃ neem oil and eucalyptus oil. Ahmed et al. [42] investigated the efficacy of powders of 4 indigenous botanicals, i.e., *Caryophyllus aromaticus* (clove), *b*lack pepper, *Trigonella foenum graecum* (methi), and neem as protectant to *C*. *chinensis* infestation in chickpea grains storage.

The current study revealed increased repellent of neem, poppy, pumpkin, and mustard oils. Abd El-Aziz & Ismail [50] reported that pumpkin oil (1% formulation) demonstrated significant repellency (88%) during the initial day which increased with increasing time. This statement promotes our findings because in the present observation, pumpkin oil showed 93.33% repellency at 2.0 ml concentration. Ratnasekera and Rajapakse [51] determined the repellency of oils and stated that vapors of oils (*C*. *nardus*, *A*. *indica*, *C*. *verum* leaf, and bark) significantly reduced *C*. *maculatus*, egg-laying, and adults’ emergence. Hanif et al. [52] determined that Datura (*Datura stramonium*), Bakain (*Melia azadarach*), and neem essential oils were highly repellent toward 3-grain storage insect pests, i.e., *Trogoderma granarium*, *Tribolium castaneum*, and *Rhyzopertha dominica*. Consequences expressed that neem was highly repellent against *T*. *castaneum* (77.66%).

Present findings recorded the highest seed germination for mustard-treated seeds, subsequently pumpkin, poppy, and neem, while the control had the lowest seed percentage. Mbaiguinam et al. [26] reported that increased rate of oils disturbed the germination ability of seeds (50%). Ramazeame et al. [53] indicated that neem-treated grains depicted an increased viability percentage than other treatments. Chelava and Khashavehb [31] noted non-significant variations for seed germination among different oils. Kumar et al. [54] reported that neem oil (2.50 ml per kg seeds) was highly effective to *C*. *chinensis*. Several studies on weed species have also suggested that extracts of various plants effectively suppress weed populations [55–60]. Therefore, these are valuable resources for pest management.

RETRACTED

## Conclusion

This study concludes that the tested oils can be employed for managing *C*. *maculatus* in stored cowpea grains. The highest concentrations of the tested oils at (i.e., 2.0 ml) were highly effective in decreasing oviposition, increasing mortality, and enhancing repellency. Neem oil performed better for inhibiting the development of *C*. *maculatus*. It is recommended the small-scale farmers or grain storage agencies must use such natural products which are not harmful to human health and environment. Further investigation for improving the effectiveness of plant-based products as insecticides will provide an advantage to the agricultural industry of developing countries.

## Supporting information

S1 Dataset The raw data used to present and interpret result in the study. (XLSX)
